RETRACTED

# Influence and Analysis of the Language and Cultural Ecological Environment in the Cognitive Process of English Writing

**DOI:** 10.1155/2022/3883459

**Published:** 2022-08-16

**Authors:** Bin Liu, Jing Wang

**Affiliations:** ^1^School of Foreign Studies, Suqian University, Jiangsu, Suqian 223800, China; ^2^School of Education, Taylor's University, Subang Jaya 47500, Selangor, Malaysia

## Abstract

Language and culture ecological environment introduces ecological theory into language and culture research, expanding the horizon of language research. The influence of language and cultural, ecological environment on English writing covers many aspects. The cognitive process of English writing involves preparation before writing, self-monitoring during writing, and self-reflection after writing. Therefore, the use of metacognition and other strategies in the cognitive process of English writing is the key to improving the cognitive level of English writing. Under the guidance of the new curriculum standards for high school English, the cognitive process of English writing should pay attention to the guidance and shaping of students' emotional experience and thinking values. Education is inseparable from the development of language and culture, and analyzing the educational ecosystem from an ecological perspective is conducive to further understanding the ecological view of language and culture. This paper focuses on the composition of the language and culture ecological environment and the influence of the language and culture environment on the cognitive process of English writing and appropriately reviews the history of cognitive psychology and ecology and development of knowledge research.

## 1. Introduction

The study of cognitive processes in English writing is of great value. Further research on the cognitive process of English writing is of great significance to English teaching [1]. Therefore, extending it to a wider perspective and field has both theoretical and practical value. Based on the connection between education and language and culture, it is feasible to integrate the cognitive process of English writing and the ecological environment of language and culture from an ecological perspective.

## 2. English Writing Cognitive Process

The cognitive process of English writing not only pays attention to the stylistic characteristics of English writing and students' English mistakes, but less research on the cognitive psychology in the writing process [2]. The cognitive paradigm in the 1980s became the dominance of Western writing psychology research, and the psychological cognitive process of writing was thus studied. Scholars have begun to pay attention to the writing process and the factors that affect writing from a cognitive perspective.

RETRACTED

### 2.1. Existing Problems in English Writing

In the 1980s, as international writing research began to turn, the process and cognitive characteristics of English writing began to be more deeply studied, and many achievements were made, but the articles on the cognitive process of English writing were extremely few. How important and complex is English writing? What strategies do English learners use to develop English writing? And what are the internal and external factors that affect English writing? Various issues are the focus areas to be studied.

Because English writing is affected by many external and internal factors, under the dual shaping of the two, the improvement of students' writing level has become the focus of research. From the perspective of writing cognitive models and metacognitive strategies, there are endless practices to improve English learners' learning level. The current new curriculum standard emphasizes knowledge, skills, emotions, attitudes, and values. However, due to cultural differences and the particularity of the language environment, students have different levels of basic language knowledge; due to the lack of metacognitive strategies and writing cognitive penetration, students ignore the value of ideas, and the layout of an article lacks certain logic. Due to the differences in language expression habits caused by cultural differences, students' English writing is deeply influenced by their mother tongue. Table 1 is the survey of Chinese college students correcting online English writing, and the results found that most college students have a low awareness of actively improving their self-writing, and their English writing is mainly for the purpose of completing homework or passing the grade.

Aiming at the problems existing in the English writing process of the above-mentioned English learners, the strategies generally adopted at present mainly include the following points. First, teachers start with cognitive strategies, analyze the root cause of learners' low writing level, and then propose relevant strategies for writing guidance. Second, urge students to strengthen the long-term memory of basic knowledge and enrich the writing cognitive database. Third, optimize the writing conception process and guide the drafting of the outline. Fourth, emphasizing review and revision to enrich students' metacognitive strategies.

### 2.2. Metacognitive Strategies

Metacognitive strategies were first proposed by American psychologist Flavell in 1976 [3]. Metacognition, that is, the individual's gradual cognitive process of oneself and the understanding of the objective existence around them can strengthen active monitoring and regulation in the process of realizing cognitive goals. Metacognition consists of three parts: knowledge, experience, and monitoring. Metacognitive knowledge is the process of constructing and learning new knowledge systems through existing schema knowledge in a specific environment; metacognitive experience is the emotional experience obtained in the process of metacognitive recognition [4]; metacognitive monitoring is the process of metacognitive monitoring. The adjustment strategy was adopted in the process.

RETRACTED

The use of metacognitive strategies in the process of English writing will greatly promote the improvement of English learning. Metacognitive strategy is an important foundation and key to helping students build a reasonable English writing knowledge system to improve their autonomous learning ability and improve their English proficiency [5]. As Figure 1 shows, metacognitive strategies are mainly reflected in the preparation before writing, the self-monitoring of the writing process, and the self-reflection and self-evaluation after writing.

English writing ability is an important output channel for comprehensive language quality and thinking ability [6]. In English writing teaching, teachers not only teach students grammar knowledge, vocabulary, and logical relationship expression and elaboration but also guide English learners to build reader awareness and enhance cultural understanding [7].

The new high school English curriculum standard “General High School English Curriculum Standard (2017 Edition)” points out that students' ability to use learning strategies is conducive to improving students' autonomous learning ability. The improvement of learning ability is not only an important content of English teaching but also an important part of the core literacy of English subjects. Writing strategy teaching is conducive to enhancing students' strategic awareness, stimulating students' interest in learning, and improving students' writing ability. Students with a high level of metacognition are better at using English writing strategies. The use of metacognitive strategies in the process of English writing is conducive to simplifying the complexity of the writing process, reducing students' fear of difficulties, and promoting students' positive cognition of English writing [8]. English writing should pay attention to the gradual progress of practical activities, design targeted activities according to students' psychological and cognitive characteristics to stimulate students' learning motivation, and personalize counseling to improve students' writing cognitive experience.

RETRACTED

### 2.3. The Cognitive Process Model and Essence of English Writing

The process-based writing model was introduced in the 1980s with oral presentations. The essence of writing is the process of psychological cognition, which is composed of the writing environment, the author's long-term memory and the writing process. The writing process and steps mainly include external factors such as writing goals, article topics, audience groups, and writing content. In addition, internal factors include the author's knowledge reserve, such as topic knowledge, rhetorical knowledge, and reader knowledge [9]. The writing process includes conception, translation, etc. The essence of reviewing is an important part of self-reflection in metacognitive strategies. Flower-Hayes's writing cognitive model breaks the one-way linear sequence of traditional writing and raises writing to a dynamic spiral repetitive process, which opens up a new field for English writing, as shown in Figure 2.

Cognitive strategies become the starting point for teachers to improve students' writing level. With the in-depth study of cognition by Flower-Hayes, the multiple factors of the writing cognition model interact, and the multifaceted interaction produces the final writing result, and the current model is different from the previous model.

Hayes' cognitive model of writing has far-reaching consequences. Many scholars have conducted more in-depth research on the psychology of writing. In Hayes's writing cognitive model, Bereto and other scholars emphasize the important value of conception in English writing [10]. The level of writing is highly related to the author's conception layout. Hayes' cognitive writing mode can be used as a staged training to guide English learners in describing the general structure of the oral composition and determining the theme of the article. In 1996, Hayes improved his original writing cognitive model and proposed a new writing cognitive model [11]. As shown in Figure 3, the research content of domestic scholars mainly focuses on conception, article layout, and word selection. Most of them recognize these factors as the key to determining the quality of articles.

## 3. The Origin of Language and Culture Ecological Environment and Its Inner Logic with Education

The concept of ecology was first proposed by the German zoologist Haeckel, and then its research principles and scope were extended to a broad perspective of linguistics and cultural studies [12]. The breadth and depth of the cognitive process of English writing depend on the richness of the writing content and the thoughtfulness of the subject. In the 1960s, cognitive psychology, in the process of changing the internal mechanism of individual information representation, the cognitive process of English writing has also been deeply studied [13].

RETRACTED

Language and culture are inseparable from education. When it comes to the language and culture ecological environment, the educational ecological environment should be mentioned.

### 3.1. Educational Environment

Any educational activity is always carried out at a certain time, in a certain place, in a certain environment, and in a certain way by certain members of the society, which reflects the constituent elements of the educational ecological environment [14, 15]. Educational ecological environment refers to the sum of all external factors that affect this educational activity as Figure 4 shows.

The natural ecological environment system refers to the natural ecological conditions in which human beings live, including abiotic factors such as topography, soil structure, water system composition, sunlight, air, minerals, and temperature, as well as biological factors such as animals, plants, and microorganisms [16, 17]. Natural ecological environment system is the foundation of human education activities, and support education activities are inseparable from the environment. The environment affects the education system, actions, and ideas between teachers and students activities within the natural ecosystem to human activity and interaction between the education provided the necessary site resources, such as education activities at the same time also provide protection for the natural ecosystem its condition, Because education can spread ecological knowledge and promote the harmonious development of human and nature, the power of knowledge enables the ecological environment to coexist with the human in a stable way. Therefore, education and the natural ecological environment have a certain dependence and positive feedback relationship.

The social and cultural environment system refers to many relationships and networks between educational activities and other social organizations as well, including values, institutional culture, traditional customs, etc. and the relationship between politics, economy, and culture [18]. The social environment of any region is a comprehensive effect on educational activities, and educational activities are an important part of the social environment [19]. As the basic engineering of society, it is not only restricted by the social environment but also reacts to the society. Social political factors, economic conditions, social and cultural customs, values, behavioral norms, scientific and technological development level, historical and cultural heritage, etc., all have an impact on educational activities and their development.

RETRACTED

Regional cultural ecosystem includes every place where students live, including school, family, community, and other ecological environments. School is the most common and effective place for students to obtain education. School facilities and atmosphere can provide a good learning environment for education. The family is the first place to receive education, and it also has a great influence on students' education.

In a word, education ecological system is a comprehensive system, education environment for students, provides a comprehensive explanation, from which we can see if the use of the content of the education of ecological system to the students' learning English writing can also create a writing for students cognitive ecosystem, all aspects of writing for the students to build cognitive training, To form a comprehensive collaborative interaction of education, cognition, and learning, so as to improve students' writing cognition.

### 3.2. Education Ecosystem

The so-called “ecosystem” refers to the functional whole composed of the biological community and the surrounding environment. The educational ecosystem is a subsystem of the ecosystem. It maintains the exchange of material, energy, and information with the natural ecology and social ecology through the cultivation of aesthetic ability. The so-called educational ecosystem refers to the educational ecological unit formed by education and other natural ecosystems, social ecosystems, etc. Through material, information circulation, and energy exchange within a certain time and space. Educational ecosystem is an educational ecosystem composed of teachers, recipients, natural environment, social environment, school environment, family environment, and other factors. It is an organic whole with certain structure and function. Through the exchange of material, energy, and information among the elements in the system, the educated person's emotion, intelligence, and personality can be developed comprehensively and harmoniously. This is the most basic function of the education ecosystem.

According to the system theory, education is a systematic project. The goals, contents, methods, means of education, teaching and receiving, etc., constitute its system structure and play a unique function of objective existence. However, the structure and function of education do not exist in isolation but have various ecological backgrounds. Local culture, customs and habits, food, and culture are all related to the goals and methods behind the educational environment, and they all influence each other. Education cannot exist independently or beyond the environment. Education itself is an ecological system, the center of which is students. The educational environment serves students, so students need to be nourished by multiple factors of the ecological environment.

RETRACTED

The educational ecosystem has rich connotations. Roughly speaking, it mainly includes the following contents: (1) “two kinds of relationships”: the relationship between people and people, and between people and the environment; (2) “three environments”: social education environment, school education environment, family education environment; (3) “four factors”: psychological factors, environmental factors, political factors, economic factors; (4) “five needs”: physiological needs, psychological needs, aesthetic needs, talent needs, and creative needs. The scientific construction of the educational ecosystem should start from these aspects so as to promote the coordinated development of various factors in the system so as to cultivate more talents needed by society as Table 2 shows.

### 3.3. Composition of Language and Culture Ecosystem

Language and its ecological environment constitute an ecological language system, which is in dynamic balance like other systems. Language is a means of communication for people in daily life and production. Cognitive as cognitive and language writing in English writing, also has its ecological system; the language in the process of English writing culture ecosystem including values, social organization, economy, science and technology; these few respects constitute the cultural ecosystem environment, under the role of cultural environment, gradually forming unique social environment and the ecological environment of language and culture. In turn, it affects the cognition of English writing. Between various factors are not independent existence at the same time; Factors exist between interdependence and mutual restriction relationship, maintaining a certain balance between various factors and is a normal material cycle and energy exchange, on the interaction relations, constituting a variety of organic connection in the nature of the whole, the so-called cultural ecology system as shown in Figure 5.

The education ecosystem can be divided into large, medium, and small, depending on how much content it contains. Large-scale education ecosystems can be at national, provincial, and regional levels, which generally describe the development laws under the background. The middle-sized one can be an ecosystem with a school or class as a unit, describing the relationship between educational and teaching policies and student development. The small educational ecosystem is the individual education system of students, which is based on students' horizontal living environment and vertical personal change or development. In short, they are representative.

RETRACTED

The educational ecosystem is diversified and omnidirectional, which has both all the factors needed by education and the influencing factors, including environment. There are both balanced development between living things and mutual construction between nonliving things, and the characteristics of their occurrence have a good guiding role for us to study the linguistic and cultural ecosystem, which provides a lot of reference and inspiration.

## 4. The Influence of Language and Cultural Ecological Environment on the Cognition of English Writing

The above analysis and overview of the cognitive mode and essence of English writing. The factors affecting the cognitive process of English writing are mainly divided into two levels: internal factors and external factors. The language and cultural ecological environment described in this paper belong to the most influential external factors. The cognitive process of English writing should be greatly influenced by its own mother tongue. Therefore, language writing has national characteristics and cultural characteristics.

In order to deeply understand the connotation of the language and culture ecological environment, this chapter expounds on the language and culture ecological environment. The language and cultural ecological environment is the environment and social and cultural environment, and its influence on language has always been widely concerned. Sapir already proposed in 1912 that according to the language people use at will, it is possible to infer the characteristics of the natural environment of the society in which they live and to remember the social and cultural characteristics [20]. This point of view is also reflected in literature, and the mutual reflection of language and social culture can be solved in literature.

The concept of language ecology was proposed by a scholar at Stanford University in the United States in 1970, which is a new perspective and milestone in the study of the relationship between language and its social environment. The language ecosystem is divided into four levels: microsystem, mesosystem, appearance system, and macrosystem. Psychological and language development is the result of the interaction of human mechanisms and the environment. This academic achievement and research perspective are highly linked to the development of cognitive psychology. Incorporating language learning into the social environment greatly expands the macroperspective of language research and gets rid of the limitations of language cognition. The language ecological environment affects the development of language characteristics, the social factors that restrict the effect of language functions, and the dynamic aggregate of the social environment. A coordinated language ecological environment can promote the generation and exertion of language and is conducive to the exertion of language functions. The internal structure of language ecological environment is intricate and complex, including the natural environment, social environment, and cultural environment related to language production and communication. The natural environment is the same as the natural environment in the educational ecological environment, and the natural environment affects the expression and representation of language. The social environment affects the communication and borrowing of languages, such as the huge number of loanwords in the Indo-European language family. The cultural environment affects the deep meaning expression of language. History and culture, ideology, ethics and values, educational science, culture, art, etc., are closely related to the cultural ecological environment of language development.

RETRACTED

Starting from the core concept of perceptual psychology and ecological psychology-permissiveness, the interaction between the language and the social environment in the language and cultural ecological environment can be analogized through the interaction between the organism and the environment in the ecosystem. Environmental properties make language full of characteristic. Vygotsky's sociocultural theory further highlights the interaction between environmental factors and learners and promotes language generation, language learning, and language communication in the interaction.

This paper mainly constructs the cognitive model of individual and environmental writing under the language and culture ecology. That is, through the language and culture ecology, the language phenomenon is placed in the ecological and cultural context, and the language generation system is regarded as an open ecosystem. In 1996, Hayes and Flower put the generation of English texts and the author's mental representation in the language ecosystem and constructed a cognitive writing model. Starting from cognitive psychology, using metacognitive strategies to cover the writing content, steps, and processes in the writing cognitive model, fully mobilize the actor's self-monitoring and self-regulation process. The revised model emphasizes the influence of macro factors such as nature, society, and culture on the cognition of English writing and examines the ecological view of language and culture from a higher level as well.

RETRACTED

The cognitive model of English writing is generated in a macroecological background. After the construction of a new cognitive model of English writing, the author summarizes the following contents of the impact of language and cultural ecological environment on English writing from practice.

First, the language and cultural ecological environment affect the vocabulary and rhetorical expressions of English writing. The generation of vocabulary involves the communication and exchange between foreign cultures, and the vocabulary of English writing will be affected by different countries and expression habit such as differences between American English and British English, including spelling and usage. Secondly, the specificity of culture will affect the rhetorical expression of language. Chinese culture is subtle and restrained, while Western culture is more unrestrained. Therefore, this cultural difference is also reflected in language rhetoric.

Second, the language and cultural ecological environment affect the thinking logic and layout of English writing. English writing pays special attention to logic, which is created by the logic of English itself. While Chinese emphasizes that the form is scattered, but the spirit is not scattered, it emphasizes the understanding of the overall meaning. Therefore, in terms of discourse layout, English is reflected in the connection between arguments and the use of logical connectives, as well as the arrangement of discourse layout. Chinese emphasizes the multiple uses of language and rhetoric.

The language and cultural ecological environment affect the basic knowledge reserve and growth of English writing. The basic knowledge of English writing varies from country to country, mainly reflected in the learning status of English in each country. For English learners in English-speaking countries, the basic knowledge of English writing is undoubtedly much higher than that in countries where English is a second or foreign language. Therefore, the cultivation of language and cultural environment is also particularly important to increase the knowledge growth and schema construction of English writing. It is necessary to strengthen the realization of long-term memory of language learners and promote the stability of basic knowledge.

## 5. Recommendations and Strategies

With the rapid development of modern society, English is becoming more and more important as the second language of most learners in the context of globalization. Learning English writing is an important part of English teaching. English writing is a learner's application of comprehensive English skills and an effective tool for students to express their ideas in writing. Many students feel that they have no idea how to write in English. Most of the students have studied English for many years, but their writing ability has not improved significantly. Many teachers also find it difficult to improve students' English writing teaching. Obviously, grammar has been taught many times, and many corresponding writing exercises have been done in class. After students have finished writing, they still do not know how to correct the grammar and sentences of the composition. Promote: As far as writing itself is concerned, the reason why students cannot complete writing well is that students have both individual problems and common problems. In view of the development of the cognitive process model of English writing, the nature of the cognitive process of English writing and the relationship between the language and cultural ecological environment, the influence of the language and cultural ecological environment on the cognition of English writing is understood. The author puts forward the following suggestions to promote the improvement of English writing effect.

RETRACTED

Firstly, according to the arrangement of the new curriculum standards for English in senior high schools, emphasis is placed on the cultivation of English learners' knowledge, skills, emotions, attitudes, and values. In the process of English teaching, it is necessary to fully understand the learning foundation of learners and the source of English writing difficulties, and then reasonably design English writing activities to stimulate the enthusiasm and initiative of learners. It is necessary to be good at adopting metacognitive strategies, enhance students' understanding of the value of strategy application, and promote their autonomous learning ability.

Secondly, we should pay attention to the creation of a language learning environment. With the help of the Internet and multimedia technology, students can experience the language charm of English-speaking countries, experience its cultural connotation, increase their emotional experience, and use literary and cultural books to cultivate students' sentiments and improve their language learning and reference ability.

Finally, we must be good at taking a variety of English writing study activities and promote the deepening of the main thought of English writing with the perception of specific situations, thereby enriching students' emotional experience. Peer assessment and collaboration through oral presentations and written results promote the application of metacognitive strategies in English writing. Create language ecology through language technology.

As can be seen from Figure 6, English writing will involve the ecological environment of the language, and the ecological environment of the language is closely related to the social environment, such as education and social culture. Therefore, infiltrating the basic knowledge of the English language and the cultural background contained in the language from literary books will improve students' learning initiative and enthusiasm while mastering the materials of English writing and then fully adopt metacognitive strategies in the writing process to complete the whole process of writing. When choosing literature books, it is necessary to determine the age of English learners and their psychological characteristics, to better combine English writing with psychological development.

RETRACTED

Language ecosystem is a narrative fable, which is suitable for use as a material reference when training narrative text writing. After fully analyzing the material, design related writing training activities to promote students' mastery of writing outlines and layout arrangements.

## Figures and Tables

**Figure 1:** The content of metacognitive strategies in the English writing process.

**Figure 2:** Hayes and Flower's cognitive model of the English writing process.

**Figure 3:** Hayes's cognitive model of writing.

**Figure 4:** The content of the natural system.

**Figure 5:** The cultural environment.

**Figure 6:** The relation between english writing and language ecosystem.

**Table 1:** The independent consciousness of Chinese college students to improve their English writing level.

Options	Subtotal	Proportion (%)
Do your own writing exercises such as English as a journal, diary, etc.	5	3.68%
Occasionally practice English writing for English grades or entrance exams	62	45.59%
Only complete the writing tasks assigned by the English teacher	65	47.79%
Do not practice English writing at all	4	2.94%
Number of valid fills in this question	136	

**Table 2:** The connotation of education ecosystem.

Two relations	Individual and individual	Individual and environment			
Three environments	Social education	School education	Home education		
Four factors	Psychological factor	Environmental factor	Political factor	Economic factor	
Five necessities	Physical need	Mental need	Aesthetic need	Development need	Creative need

## Data Availability

The labeled dataset used to support the findings of this study is available from the corresponding author upon request.
